The article "The Effect of Different Treatment Methods on Acute Acquired Concomitant Esotropia" was retracted in 2023. Reasons: signs of a paper mill; suspected computer-generated content; unreliable results or conclusions; concerns about the data.

# The Effect of Different Treatment Methods on Acute Acquired Concomitant Esotropia

**DOI:** 10.1155/2022/5001594

**Published:** 2022-04-23

**Authors:** Xiaoqi Huang, Yanfang Meng, Xuemin Hu, Yijia Zhao, Meihong Ye, Beixi Yi, Lianhong Zhou

**Affiliations:** Department of Ophthalmology, Renmin Hospital of Wuhan University, Wuhan 430060, China

## Abstract

**Objective:**

The application of botulinum toxin type A (BTXA) in the treatment of paralytic strabismus has been recognized, but there are few studies on the treatment of acute acquired comitant esotropia (AACE). This study was aimed to investigate the clinical characteristics of AACE and compare the therapeutic effects of BTXA and traditional surgery.

**Methods:**

78 patients with AACE in Renmin Hospital of Wuhan University between March 2019 and March 2021 were reviewed. The relevant medical records of the patients were collected, and they were divided into surgical group (*n* = 46) and botulinum toxin type A (BTXA) group (*n* = 32) according to different treatment approaches. The surgical group was treated with squint correction, whereas the BTXA group was treated with microinjection of BTXA in MR. Eye alignment, esotropia, stereopsis, and complications were examined before and after treatment in both groups.

**Results:**

The refractive status of 78 patients with AACE was mostly myopic refractive error. In general, the angle of esotropia at distance was larger than which at near, with a statistically significant difference. At follow-up assessments of 1 week, 1 month, 3 months, and 6 months after treatment, the total effective rates of the surgical group and the BTXA group were 100% and 90.48%, respectively. The residual angle of esotropia of both groups was lower after treatment. Additionally, the incidence rate of complications in the BTXA group was significantly lower than that in the surgical group.

**Conclusion:**

AACE occurs mostly in people with myopic refractive errors and is associated with prolonged near work. Besides surgical treatment, micro-injection of BTXA is also an effective and safe treatment for AACE.

## 1. Introduction

Acute acquired comitant esotropia (AACE) is a specific type of strabismus which occurs in older children and adults [1]. AACE is generally considered a relatively rare type of strabismus, accounting for approximately only 0.3% of patients with strabismus [2], which has a rapid onset and generally late onset [3]. It is characterized by sudden onset constant esotropia with diplopia, but there are no abnormalities in the neurological system [4]. AACE is classified into three types according to the clinical characteristics and etiologies by Burian and Miller [5]: Swan type (type 1), which has a sudden onset due to interrupted fusion by monocular occlusion or vision loss; Burian–Franceschetti type (type 2), which may be caused by physical or psychological stress and is demonstrated by large deviations, small refractive errors, and minimal accommodation; and Bielschowsky type (type 3), which is associated with moderated myopia or might result from excessive near work activities [2]. However, in recent years, with the popularity of electronic products such as IPads and smartphones and the increased academic pressure on students, the incidence of AACE has been on the rise [6]. The etiology of AACE is still unclear, which may be related to the destruction of binocular fusion function, original cryptostrabismus or myopic ametropia, or the anatomical abnormality of medial rectus muscle or nervous system abnormality [1].

Currently, common treatments for AACE include wearing prism, surgery of squint correction, and microscopic medial rectus muscle injection of botulinum toxin type A (BTXA) [7]. BTXA is a neurotoxin produced by Gram-positive anaerobic bacteria, which has the effect of muscle paralysis [8]. After a series of reactions, BTXA inhibits the release of the neurotransmitter acetylcholine at the neuromuscular junction, resulting in muscle paralysis [9]. In 1981, Scott [10], an American physician, first proposed that BTXA had the effect of extraocular muscle paralysis, and it was first used in clinical strabismus treatment. When BTXA was injected into the medial rectus muscle of the non-dominant eye of AACE patients, the muscle strength of the injected muscle was weakened for a period of time so that the muscle strength of the affected eye could be rebalanced, thus achieving the purpose of correcting eye position and disappearing diplopia [11]. BTXA injection for AACE is less expensive than surgery, and the operation is simple and fast and has fewer complications such as intraoperative bleeding and postoperative infection. Moreover, the toxin has no long-term ocular or systemic side effects when injected into the extraocular muscles, and repeated injections are not recognized by the immune system, so there is no allergic reaction [12]. Nevertheless, BTXA injection for AACE also has some limitations, such as limited duration of drug action and the occurrence of adverse reactions.

This study collected medical records of 78 patients with AACE in Renmin Hospital of Wuhan University between March 2019 and March 2021, aiming to explore the clinical characteristics of AACE and to compare the therapeutic effects of BTXA and surgery of squint correction for AACE.

## 2. Materials and Methods

### 2.1. General Information

The medical records of all patients with AACE at the Ophthalmology Center, Renmin Hospital of Wuhan University from March 2019 to March 2021 were followed up for more than 3 months and were reviewed.

In total, 78 cases fulfilled the inclusion criteria, including 46 cases treated with surgery and 32 cases treated with BTXA injection. All patients were subjected to follow-up assessment at 1 week, 1 month, 3 months, and 6 months after treatment to observe and compare eye alignment, angle of esotropia deviation, diplopia, eye movements, stereopsis, and any presenting complications.

Inclusion criteria are as follows: (1) acute onset of comitant esotropia with diplopia; (2) no strabismus before onset; (3) same deviation in all gaze directions (deviation difference< 5PD); (4) no limited eye movement; (5) no abnormality in neurological system; (6) corrected visual acuity of 6/6 in both eyes; and (7) follow-up time> 3 months.

Exclusion criteria are as follows: Patients with a history of eye diseases, including paralytic strabismus, previous ocular trauma, previous ocular surgery and amblyopia, with neurological diseases such as pituitary tumor, and myasthenia gravis were excluded.

The study adhered to the tenets of the Declaration of Helsinki and was approved by the Ethics Committee of Renmin Hospital of Wuhan University. The need for individual informed consent was waived by the ethics committee because of the retrospective nature of the study.

### 2.2. Methods

Basic information about patients was obtained, including (1) gender, age, occupation, and daily duration of near work; (2) course and duration of onset; (3) history of previous ocular diseases, surgery, and trauma; and (4) systemic conditions, including those affecting the neurological and endocrine systems.

Routine ophthalmic examinations were performed in all patients before treatment, including visual acuity (best corrected visual acuity), cycloplegic refraction, slit-lamp assessment of the anterior segment, intraocular tension, deviation at near and distance fixation, and stereoacuity. Cycloplegic refraction measurement was performed after the instillation of 1% atropine ointment twice daily for five days in patients under 12 years old and 1% cyclopentolate eye drops every five minutes three times in patients over 12 years old. Spherical equivalents (SE) of refractive error were calculated using the algebraic sum of the dioptric powers of the sphere and half of the cylinder. An oculomotor examination was performed to determine whether the eye movement was limited. Ocular motility and nystagmus were evaluated clinically. The angle of deviation was measured with the triangular prism and alternate cover tests at 33 cm (near) and 6 m (distance) fixation. Stereoacuity was assessed with the Titmus test card at 40 cm.

All patients underwent ophthalmic and orthoptic examinations, cranial and orbital computed tomography (CT), or magnetic resonance imaging (MRI) to exclude neurological diseases and thyroid function tests and endocrinology consultation to exclude endocrine system diseases such as hyperthyroidism.

### 2.3. Treatments

Surgery of strabismus correction (surgical group (*n* = 46)): patients with the onset of AACE for more than 6 months, a large degree of deviation, diplopia symptoms seriously affecting the quality of life, or conservative treatment failed. The design of the surgical operation was as follows: Unilateral medial rectus muscle recession was performed in 4 cases with ≤ +20^△^; medial rectus muscle recession and lateral rectus muscle resection was performed in 39 cases with +20^△^~+60^△^; and bilateral medial rectus muscle recession combined with unilateral or bilateral lateral rectus muscle resection in 4 cases with >60^△^. The operation process is as follows: (1) select the appropriate anesthesia method according to the patient's age; (2) after successful anesthesia, routine disinfection and towel laying were carried out; (3) 0.5% Alcaine was used for topical anesthesia, and 0.01% epinephrine hydrochloride was used for vasoconstriction; (4) 2% lidocaine hydrochloride was injected for subconjunctival infiltration anesthesia; (5) the conjunctive incision near the fornix was made on the corresponding nasal or temporal bulbar conjunctiva of the operated eye to separate the intermuscular membrane and subconjunctival tissue and fully expose the medial rectus muscle and lateral rectus muscle; (6) double looped sutures were used at the insertion of rectus muscle for medial rectus recession or lateral rectus shortening; and (7) continuous suture of bulbar conjunctiva. In cases with local anesthesia, the sutures can be adjusted intraoperatively according to the eye position and corneal optical reflection to achieve the alignment. For patients with general anesthesia surgery, the surgical effect may be slightly worse than that of patients with local anesthesia because the intraoperative eye position cannot be observed and adjusted.

Microscopic medial rectus muscle injection of BTXA (BTXA group (*n* = 32)): patients with onset of AACE for more than 6 months, ineffective conservative treatment and refusal of strabismus correction. The dosage of BTXA was selected as follows [13]: 1.0 U~2.5 U for those < +20^△^, 8 cases; 2.0 U ~ 4.0 U for those from +20^△^ to +40^△^, 23 cases; and 4.0 U ~ 6.0 U for those > +40^△^, 7 cases. The maximum dosage of each muscle did not exceed 5 U, and the total volume of injection every time did not exceed 0.1 mL. The injection procedure was as follows: (1) The eyelid opener was used to open the eye, and 0.5% Alcaine was used for topical anesthesia, and 0.01% epinephrine hydrochloride was used for vasoconstriction; (2) 2% lidocaine hydrochloride was injected for subconjunctival infiltration anesthesia; (3) made a conjunctival incision near the bulbar conjunctiva on the nasal side of the operated eye, then the medial rectus muscle was hooked, and the intermuscular membrane and subconjunctival tissue were separated to fully expose the medial rectus muscle; (4) the botulinum toxin type A (BTXA) was dissolved in an appropriate amount of sterile saline to configure the required dose of solution; and (5) corresponding dose of botulinum toxin type A (BTXA) was injected intramuscularly at 5 mm from the muscle insertion (the total amount of each injection should not exceed 0.1 mL).

### 2.4. Curative Criteria

The patients complained that diplopia disappeared and the angle of residual deviation <10^△^ (measured with the triangular prism and alternate cover tests).

### 2.5. Statistical Analysis

SPSS version 25.0 (SPSS Inc., Chicago, IL, USA) was used for statistical analysis. Continuous variables are presented as mean ± standard deviation (SD). Continuous non-normal distribution variables are represented as median and interquartile. The enumeration data between groups were compared by a chi-square test. The measurement data between groups were compared by independent *t*-test. The Friedman test was used to compare the degree of deviation angle before and after treatment within each group. The Wilcoxon signed rank test was used to compare the efficacy between the surgical group and the BTXA group, as well as to compare the deviation at near and distance fixation. Fisher's precision probability test was used to compare the efficacy of the two groups. Cochran's Q test was used to compare stereoscopic results across different times. *P* values < 0.05 were considered statistically significant.

## 3. Results

### 3.1. Characteristics of the Patients

A total of 78 AACE patients were included in this study (Table 1). The mean onset duration was 21.81 ± 8.64 months (from 6 to 120 months). Most patients reported working in close proximity (< 33 cm) for long periods of time before onset. The mean duration of daily near work before onset was 8.58 ± 1.65 hours (from 4.5 to 12 hours). Among them, 55 patients (70.51%) spent more than 8 hours near work daily, but only 23 patients (29.49%) spent less than 8 hours daily. None of the patients had a family history of strabismus, trauma, and occlusion of one eye. External and anterior segments were normal in all patients.

Eye movements in all gaze directions had no limitations. Ocular examinations and neurological examinations were normal in all patients. The follow-up duration was at least 3 months.

When the general conditions of the two groups of patients were compared in terms of gender, age, duration of daily near work, duration of onset, and SE, no statistically significant differences were found (*P* > 0.05), indicating that there was comparability between the surgical group and BTXA group (Table 2).

### 3.2. Comparison of Deviation Angle at Distance and near

The angle of deviation was +20^△^ (+12^△^ to +98^△^) at near (33 cm) and+ 25^△^ (+16^△^ to +96^△^) at distance (6 m) fixation. Among the 78 cases, 52 cases presented a deviation at distance fixation larger than that at near fixation. 18 cases presented the deviation at distance fixation less than that at near fixation. The other 8 patients had the same deviation at both near and distance fixation. The overall deviation of AACE patients at distance fixation was larger than that at near fixation, and the difference was statistically significant (*Z* = −5.560, *P* < 0.05, Table 3).

### 3.3. Comparison of Deviation before and after Treatment in each Group

At follow-up assessments of 1 week, 1 month, 3 months, and 6 months after treatment, the deviation angle at near and distance in the two groups were compared, respectively. A statistically significant difference (*P* < 0.05) was found between the two groups in terms of near (30 cm) and distance (6 m) at pretreatment and 1-week posttreatment. The deviation angle of patients in the BTXA group was significantly smaller than that of the surgical group before and 1 week after treatment. One week after treatment, there was a significant difference in the deviation angle between the two groups. It is because some patients in the BTXA group had overcorrection due to the early effect of the drug, which disappeared with the prolongation of the drug effect and the eye alignment gradually returned to orthotropia. The differences were not statistically significant (*P* > 0.05) when comparing the deviation angle in the two groups at 1, 3, and 6 months posttreatment follow-up, indicating that the efficacy of the two treatment modalities was equivalent in the long term (Figures 1(a) and 1(b)).

### 3.4. Comparison of Therapeutic Effects in the Surgical and BTXA Groups

After 6 months follow-up, the orthotropia rate was 97.82% in the surgical group and 90.63% in the BTXA group (Table 4). Three patients in the BTXA group had recurrence of deviation in two weeks, one month, and three months after treatment, and they complained of diplopia again, and the angle of deviation was more than +10^△^. In one case, the original deviation degrees were both +25^△^ at near (33 cm) and distance (6 m), and the postrelapse deviation degrees were both +16^△^ at near (33 cm) and distance (6 m). The remaining two cases had the same postrelapse deviation degree as before. However, comparing the total efficiency (at near and distance) of the two treatments, no statistically significant differences were found (at near: *Z* = −0.018, *P* > 0.05; at distance: *Z* = −0.761, *P* > 0.05).

### 3.5. Comparison of Stereoacuity in the Surgical and BTXA Groups

Before treatment, a comparison of the stereopsis of patients in the surgical and BTXA groups revealed no statistically significant difference (*χ*^2^ = 0.851, *P* > 0.05). At the follow-up from 1 week to 6 months after treatment, the differences were still not statistically significant (*P* > 0.05).

In the surgical group, the proportion of patients with stereoscopic function before surgery, 1 week, 1 month, 3 months, and 6 months after surgery was 63.0%, 80.4%, 87.0%, 93.5%, and 93.5%, respectively. The difference of stereoscopic function at 5 follow-up assessments was statistically significant (Cochran's *Q* = 39.765, *P* < 0.05).

In the BTXA group, the proportion of patients with stereoscopic function before injection, 1 week, 1 month, 3 months, and 6 months after injection was 65.6%, 75.0%, 84.4%, 90.6%, and 90.6%, respectively. The difference of stereoscopic function at 5 follow-up assessments was statistically significant (Cochran's Q = 22.857, *P* < 0.05).

Five follow-up assessments before and after treatment revealed that the stereoscopic function improved after treatment compared to pretreatment, both with surgery and BTXA injection: The number of patients without stereopsis (> 800″) decreased, and the number of patients with peripheral stereopsis (300″ ~ 800″), macular stereopsis (70″ ~ 200″), and foveal stereopsis (≤ 60″) increased, with statistically significant differences (*P* < 0.05) (Table 5).

### 3.6. Comparison of Complications in the Surgical and BTXA Groups

There are different complications in both two treatments (Table 6). In the surgical group, 9 postoperative complications of subconjunctival hemorrhage occurred. In the BTXA group, one case of vertical strabismus and 3 cases of ocular motility restriction were observed. The complications of the two groups were short-term complications, and there were no special complications in the two groups after long-term observation. Although the complication rate of treatment in the BTXA group was lower than that of the surgical group (19.57% *vs*. 12.5%), there was no statistical difference (*P* > 0.05).

## 4. Discussion

AACE is a sudden and specific type of esotropia, which mostly occurs in older children and adults [14]. It is characterized by a sudden onset of concomitant esotropia with approximately the same degree of deviation in all fields of gaze, accompanied by diplopia, and no limitation of eye movement [15]. Lee et al. [6] in 2016 found that adolescents with myopia, mild hyperopia, or normal vision (i.e., susceptible population) may develop AACE after excessive smartphone use at close range. Avoiding the use of smart phones may reduce the degree of deviation in patients with AACE, and the residual deviation may also be successfully corrected by surgery. In this study, we collected the duration of near work before onset in 78 patients and found that more than half (70.51%) patients had a daily average duration of near work of more than 8 h before onset. Prolonged near work results in vergence overuse, which increases the tension of the medial rectus muscle; then, AACE occurs when the force of separation is insufficient to overcome the force of assembly.

Buch and Vinding [16] divided AACE into four types based on Burian's study [5]: Type IV, which is postoperative loss of compensation; Type V, which is associated with intracranial disease and neurological manifestations; Type VI, which is AACE manifested as periodic esotropia; and Type VII, which is AACE combined with other ocular diseases. KOTHARI also added two new types to the original typology [17]: Type IV, also known as refractive adjustment type, is characterized by the presence of high hyperopia, and the degree of deviation and diplopia can be controlled after hyperopia correction, and Type V, also known as cranial fossa lesion-related type, is an AACE combined with intracranial lesions, especially posterior cranial fossa-related lesions. However, the common clinical typology is still the first three classical types summarized by Burian and Miller above. In this study, among the 78 cases of AACE, 65 cases were myopia, accounting for 83.33%. The mean spherical equivalent of 78 patients with AACE was −3.77D ± 3.13D of the right eyes and −3.69D ± 3.23D of the left eyes, which indicates that the 78 cases of AACE in this study were mostly type III.

The surgical outcomes of AACE are not yet established as most previous reports studied a few patients at various ages. Strabismus correction is a microscopic procedure in which the patient's eye position is corrected and diplopia disappears by means of medial rectus muscle recession and lateral rectus muscle resection. It is generally used for patients with a large degree of deviation or patients who have failed conservative treatment [18]. The timing of surgery is generally chosen when the deviation is relatively stable after more than 6 months of conservative treatment [19]. All 46 surgical patients in this study had an onset of more than 6 months, were ineffective in conservative treatment, and underwent surgery when their deviation was more stable.

The most frequent side effect caused by extraocular muscle injections of BTXA is ptosis [7], due to the diffusion of BTXA into the adjacent muscles of the eye, especially the levator muscle, which is relatively sensitive to BTXA. Among the 32 patients who opted for BTXA injections in this study, 29 had an orthotropic eye position at the last follow-up, and 3 patients exceeded the duration of action of BTXA and had a recurrence of deviation. Three patients who had a recurrence were offered the choice of another BTXA injection or the choice of surgery. Three patients chose surgery, and one patient chose a second BTXA injection for treatment. In the 32 AACE patients in the BTXA group, three patients had limited eye movement on the second day after injection, which was manifested as slightly limited movement of the affected eye in the nasal direction, and this symptom disappeared at the later follow-up. It may be due to the denervation of the internal rectus muscle injected with BTXA, and the denervation also affected the spouse muscle of this muscle, which eventually resulted in mild limitation of movement, the exact cause of which needs to be further investigated. One patient showed mild vertical strabismus at follow-up 1 week after injection, and these symptoms of vertical strabismus disappeared by the follow-up visit one month later. The remaining patients presented with no special symptoms, and self-reported symptoms were good at the final follow-up visit.

In general, after 3 months of follow-up, the residual deviations of the two groups after treatment were lower than those before. Comparing the total orthotropia rate (at near and distance) of the surgical group and the BTXA group, no statistically significant difference was found, which showed that both surgical and BTXA injection for AACE could achieve the purpose of alleviating the degree of deviation and diplopia. In addition, the results showed that the incidence of postoperative complications in the BTXA group was lower than that in the surgical group, but the overall difference in postoperative complications between the two groups was not statistically significant, indicating that the safety of BTXA injection for AACE was comparable to that of surgery. Lang et al. also found that the therapeutic effect of botulinum toxin injection on AACE is similar to that of squint correction and the procedure is simpler in botulinum toxin injection than in squint correction [11]. Therefore, botulinum toxin injection may be a good choice for treatment of AACE.

However, there are some limitations to BTXA injection for ACCE, such as the limited duration of action of the drug. After injection of BTXA, efficacy disappeared for a period of time in some patients, eye position will change, and there will be a certain degree of recurrence of deviation, or even back to the initial deviation. The patients with recurrence of esotropia can choose to have a second injection of BTXA, or they can choose surgical treatment. Therefore, in future clinical work, we will continue to collect typical cases, expand the sample size, and conduct comparative studies.

## 5. Conclusion

In summary, AACE occurs mostly in people with myopic refractive errors and is associated with prolonged near work, especially the excessive use of electronic devices such as smartphones and tablet computers. For patients with larger angle of deviation and ineffective conservative treatment, in addition to the commonly used surgical treatment, microscopic injection of BTXA for AACE is also an effective and safe treatment, which has been widely used in clinical practice. In general, there was no statistically significant difference in the incidence of complications between the two treatments.

## Figures and Tables

**Figure 1:** Comparison of deviation before and after treatment in each group. The angle of deviation was measured with the triangular prism and alternate cover tests at 33 cm (near, a) and 6 m (distance, b) fixation. BTXA, botulinum toxin type A. Data was expressed mean ± SD. ∗*P* < 0.05; ns, no significant difference.

**Table 1:** Clinical characteristics of AACE patients.

Variables	*N* = 78
Gender (male: female)	50 : 28
Age at onset (years)	30.14 ± 10.36
Duration of onset (months)	21.81 ± 8.64
Spherical equivalent (diopter)	
Right	−3.77 ± 3.13
Left	−3.69 ± 3.23
Duration of daily near work (hours)	8.58 ± 1.65
< 8 hours	23 (29.49%)
≥ 8 hours	55 (70.51%)
The angle of esotropia deviation pre-injection (PD^a^)	
Near	+31.58 ± 17.25
Distance	+35.68 ± 17.32
Stereoacuity pre-injection	
Stereopsis (+)	50 (64.10%)
Stereopsis (-)	28(35.90%)

^a^ PD: prism diopters.

**Table 2:** Comparison of clinical data of AACE patients with different treatments.

Group	Sample (n)	Gender (*n*)		Age (year)	Daily near work (hour)	Onset duration (month)	Spherical equivalent (diopter)	
		Male	Female				OD	OS
Surgical	46	31	15	29.89 ± 10.11	8.50 ± 1.44	21.10 ± 14.37	−3.20 ± 3.40	−3.09 ± 3.34
BTXA	32	19	13	29.90 ± 10.86	8.67 ± 1.92	22.68 ± 15.71	−4.60 ± 2.52	−4.56 ± 3.89
*t*/*χ*2		0.527		-0.605	-0.564	-0.138	0.290	0.109
*P*		0.468		0.549	0.576	0.450	0.107	0.554

**Table 3:** Comparison of deviation angle at near and distance.

Type of deviation angle	Sample (*n*)	*Z*	*P*
Near < distance	52		
Near = distance	18	-5.56	<0.05
Near >distance	8		

**Table 4:** Comparison of therapeutic effects in surgical and BTXA groups.

Distance	Treatment	Sample (*n*)	Diplopia (*n*)	Follow-up deviation (*n*)		*Z*	*P*
				< 10 PD	≥10PD		
33 cm	Surgery	46	1	45	1	-0.018	>0.05
	BTXA	32	3	29	3		
6 m	Surgery	46	1	45	1	-0.761	>0.05
	BTXA	32	3	29	3		

**Table 5:** Comparison of stereoacuity in surgical and BTXA groups.

Times	Group	Stereoacuity			
		No^a^	Peripheral^b^	Macular^c^	Central concave^d^
Pre-injection	Surgical	17	15	13	1
	BTXA	11	10	9	2
Post-injection					
1 week	Surgical	9	18	16	3
	BTXA	8	10	11	3
1 month	Surgical	6	14	20	6
	BTXA	5	9	14	4
3 months	Surgical	3	16	20	7
	BTXA	3	10	14	5
6 months	Surgical	3	17	19	7
	BTXA	3	11	12	6

^a^No: no stereopsis (> 800″). ^b^Peripheral: peripheral stereopsis (300″~800″).^c^Macular: macular stereopsis (70″~ 200″). ^d^Central concave: central concave stereopsis (≤ 60″).

**Table 6:** Comparison of complications in the surgical and BTXA groups.

Group	Sample (*n*)	Complications			Total (*n*)	Incidence (%)	*χ*2	*P*
		Subconjunctival hemorrhage	Vertical strabismus	Limitation of eye movement				
Surgical	46	9	0	0	9	19.57	0.018	>0.05
BTXA	32	0	1	3	4	12.50		

## Data Availability

The data used to support the findings of this study are available from the corresponding author upon request.
